The article "The Indices of Instantaneous Pulse Rate Variability Are Indicators for Daily Life Quality Assessment in Patients with COPD" was published in 2022. Journal: J Healthc Eng.

# The Indices of Instantaneous Pulse Rate Variability Are Indicators for Daily Life Quality Assessment in Patients with COPD

**DOI:** 10.1155/2022/6103305

**Published:** 2022-02-10

**Authors:** Po-Hsun Huang, Yi-Fei Luo, Tzu-Chien Hsiao

**Affiliations:** ^1^Institute of Computer Science and Engineering, College of Computer Science, National Yang Ming Chiao Tung University, Hsinchu, Taiwan; ^2^Service Systems Technology Center, Industrial Technology Research Institute, Hsinchu, Taiwan; ^3^Department of Computer Science, College of Computer Science, National Yang Ming Chiao Tung University, Hsinchu, Taiwan; ^4^Institute of Biomedical Engineering, College of Electrical and Computer Engineering, National Chiao Tung University, Hsinchu, Taiwan

## Abstract

Chronic obstructive pulmonary disease (COPD) is a progressive respiratory illness. Questionnaires such as modified Medical Research Council (mMRC) dyspnea scale and COPD assessment test (CAT) are useful for COPD condition and life quality assessment. These questionnaires reflect how respiratory disorder affects daily life. Breathing and autonomic nervous system (ANS) usually regulate each other. Few studies discussed the ANS activity and daily life quality in patients with COPD. Therefore, this study aimed to find the relationship between daily life quality assessed by mMRC or CAT and ANS assessed by a novel method, instantaneous pulse rate variability (iPRV), a method indicating not only the ANS activity but also the peripheral response. The result showed that the change in mMRC and the change in low frequency power to high frequency power ratio, which usually represents the sympathetic activity in conventional heart rate variability analysis, had significant correlation (*r* = 0.63; *p* < 0.05). The change in CAT and the change in high frequency power (regulated by vagal nervous and respiratory system) or very high frequency power (new frequency band can be indicated in iPRV spectrum) had significant negative correlation (*r* = −0.64 and −0.55, respectively; *p* < 0.05 for both). This study showed the change in iPRV indices when the condition of COPD was improvement or exacerbation. This study presents a possible way to show how cardiovascular activity affects daily life quality in patients with COPD. Increase in LF or decrease in HF and VHF would cause poorer quality of daily life in patients with COPD. The result can also be a reference for patients with COPD to choose the breathing type to adjust rehabilitation and therapy program for ANS regulation to indicate or improve their daily life quality.

## 1. Introduction

Chronic obstructive pulmonary disease (COPD) is a complex disorder of lung tissue which leads to airflow limitation. COPD is also a common progressive illness which causes long-term breathing problem. The main symptoms of COPD include cough and shorter breathing. In clinic, the forced vital capacity (FVC) and the forced expiratory volume in one second (FEV1) are usually measured by spirometer for COPD diagnosis. The ratio between FEV1 and FVC is usually lower than 70% in the patients with COPD [1, 2]. Additionally, questionnaires such as modified Medical Research Council (mMRC) dyspnea scale and COPD assessment test (CAT) are also useful for the COPD diagnosis [3, 4]. These two questionnaires are widely used in clinic for investigating the life quality of patients with COPD. Medical Research Council dyspnea scale (MRC) was first described by Fletcher [5] to assess the breathlessness in patients with emphysema. According to the patients' ability to perform physical activities, five grades (from 1 to 5) in MRC were used for quantification. Previous research showed the usefulness of MRC as a measure of disability in patients with COPD. The modified version of MRC (mMRC) is used today. mMRC modified the statement to be simpler; it also contains five stages of breathlessness according to physical exertion (from 0 to 4). CAT was proposed by Jones et al. in 2009 for providing a short, simple, and reliable questionnaire to monitor COPD [3]. There are eight candidate items in CAT for assessing the influence between symptoms and impacts of COPD. The results of mMRC and CAT have shown the relationship with the severity of COPD [1, 6–10]. According to Global Initiative for Chronic Obstructive Lung Disease (GOLD), the result of mMRC or CAT and spirometry can help us separate the patients with COPD into different severity groups (GOLD A, GOLD B, GOLD C, and GOLD D).

The article "The Indices of Instantaneous Pulse Rate Variability Are Indicators for Daily Life Quality Assessment in Patients with COPD" was published in 2022. Journal: J Healthc Eng.

COPD might influence the patients' respiratory mechanism. Moreover, research showed that the patients with COPD also have higher risk of suffering from cardiovascular disease (CVD) [11]. The study showed the respiratory activity might have relation to the cardiovascular activity. For the cardiovascular assessment, the autonomic nervous system (ANS) indication is needed. The ANS, including sympathetic nervous system (SNS) and parasympathetic nervous system (PNS), regulates our body's unconscious actions. The heart activity and vasoconstriction or vasodilation are dominated by ANS. For example, SNS stimulates the heart for higher heart rate. In contrast, PNS makes heart rate decrease. For indicating the activity of ANS, heart rate variability (HRV) is one of the useful noninvasive methods [12]. The R-peak of electrocardiogram (ECG) is used for HRV calculation. After the R-R interval (RRi) series calculation, the time domain analysis (e.g., SDNN) or frequency domain analysis (e.g., low frequency power) can be performed for further analysis. Volterrani et al. found HRV decrease in COPD group compared with normal group [13]. Some studies also showed the difference in HRV under different breathing maneuver [14–16] or the correlation between HRV indices and other measurements [15–17]. Kabbach et al. also found the higher modulation of PNS in COPD exacerbated patients [18].

However, the time resolution of RRi limits the research of HRV. In frequency domain analysis of HRV, the meaningful frequency band power can only be found under 0.5 Hz [19]. A novel method called instantaneous pulse rate variability (iPRV) was proposed for breaking the limitation [20]. iPRV is calculated from photoplethysmography (PPG) or atrial blood pressure (ABP) instead of ECG. Though the pulse arrival time (PAT) exists between the P-wave and R-peak, PPG-based HRV (or called pulse rate variability, PRV) can be still a surrogate for ECG-based HRV [21]. Previous studies also showed the similar result between HRV and iPRV in conventional indices under different situations [20, 22, 23]. iPRV applies the Hilbert–Huang transform technique to break the resolution limitation of HRV.  Figure 1 (left) shows that the time resolution of iPR series is much higher than the RRi. Extra information can be found in iPRV power spectrum (on the right of Figure 1). The very high frequency (VHF) band which is the frequency band higher than conventional high frequency band in HRV is also indicated in the iPRV power spectrum.

Previous research showed the correlation between spirometry indices and HRV indices [16, 17]. However, fewer studies compared the details of mMRC or CAT with the HRV indices. Moreover, fewer studies compared the points change in mMRC or CAT of the patients with COPD with condition improvement or exacerbation. These two questionnaires are important for daily life quality assessment of patients with COPD. In addition, the novel indices calculated by iPRV can be also compared with the questionnaires. Some studies showed that VHF calculated by iPRV had possible meaning of peripheral response [24]. Therefore, the aim of this study was to measure mMRC, CAT, and iPRV indices two times to find the correlation between the mMRC or CAT and iPRV indices. We try to find how cardiovascular activity, peripheral response, and breathing problem affect the daily life quality in patients with COPD.

## 2. Materials and Methods

### 2.1. Study Design

In this study, the patients with COPD participated in the experiment in two phases, phase A and phase B. In each phase, the experiment was conducted twice, and the second time was one week after the first time. The second experiment result in each phase was used in this study because we assume that the subjects would be more familiar with the experiment procedure and measurement. Phase B experiment was carried out at least two months after phase A. The vital capacity at a sampling rate of 556 Hz, respiratory inductive plethysmography at a sampling rate of 32 Hz, and PPG signal at a sampling rate of 128 Hz were measured at the same time in each experiment. The subjects were asked to follow standard procedure of vital capacity measurement in the first minute. The subjects were asked to do spontaneous breathing in the following five minutes. The subjects were in sitting position during signal acquisition. The stable ninety seconds of PPG signal of the last five minutes were used for iPRV analysis in this study. The mMRC, CAT, and lung function test results were collected from medical record provided by the patients. The experiment was performed in the Taipei Veterans General Hospital, Taiwan. Informed consent was obtained from all subjects before the experiment.

The article "The Indices of Instantaneous Pulse Rate Variability Are Indicators for Daily Life Quality Assessment in Patients with COPD" was published in 2022. Journal: J Healthc Eng.

### 2.2. Subjects

14 subjects who were diagnosed with COPD by doctors were enrolled in this study. The ratio between FEV1 and FVC of all subjects was lower than 70%. The basic information of subjects is shown in Table 1. Between phase A and phase B, subjects regularly came back to hospital every month. The patients' status was checked by doctors to confirm that the patients were suitable for this study.

### 2.3. Lung Function and Questionnaires

The lung function test and questionnaires were measured by doctors. The patients provided their medical records for this study.

### 2.4. iPRV Procedure

The PPG signals were used for calculating the iPRV. The iPRV applies the decomposition technique of HHT called empirical mode decomposition (EMD) to decompose the PPG signal into intrinsic mode functions (IMFs) [25]. The IMFs satisfy two conditions: (1) the number of local minimum and local maximum must be equal to the number of zero-crossings or differ at most by one, and (2) the value of average envelop must be approximately equal to zero at any point. The EMD procedure for finding the IMF is as follows: Let *x(t)* denote the original input signal and *xi(t)* denote the *i*th input after (*i*-1)th IMF is extracted. The first step of EMD is to find the local maximum and local minimum of the input signal *x*_*i*_*(t)* to calculate the upper envelope *U(t)* and lower envelope *L(t)*. We can calculate the average envelope by average *U(t)* and *L(t)*:

(1) $$\begin{array}{c} \text{M}\left(\text{t}\right)=\frac{\text{U}\left(\text{t}\right)+\text{L}\left(\text{t}\right)}{2}, \end{array}$$

and the output of this iteration can be

(2) $$\begin{array}{c} \text{H}\left(\text{t}\right)={\text{x}}_{\text{i}}\left(\text{t}\right)-\text{M}\left(\text{t}\right). \end{array}$$

The above process is called sifting processing. Then, judge whether the *H(t)* is IMF or not. If *H(t)* is not an IMF, let *H(t)* be the input to the next iteration of the sifting processing until the *H(t)* is an IMF. If *H(t)* is an IMF, output *H(t)* as the IMF *c*_*i*_*(t)* and let the residual *r(t)* of *x*_*i*_*(t)* be the input *x*_*i+1*_*(t)* to the next iteration of the above steps.

(3) $$\begin{array}{c} \text{r}\left(\text{t}\right)={\text{x}}_{\text{i}}\left(\text{t}\right)-{\text{c}}_{\text{i}}\left(\text{t}\right), \end{array}$$

(4) $$\begin{array}{c} {\text{x}}_{\text{i}+1}\left(\text{t}\right)=\text{r}\left(\text{t}\right). \end{array}$$

Redo the above steps until *x*_*i+1*_*(t)* is a monocomponent. For avoiding mode mixing problem, complete ensemble EMD (CEEMD) [26] was used in this study. CEEMD adds white noise *N(t)* described as follows to the original input signal *x(t)* to eliminate the mode mixing.

(5) $$\begin{array}{c} \left[\begin{array}{c} {\text{x}}_{\text{p}}\left(t\right)\\ {\text{x}}_{\text{n}}\left(t\right) \end{array}\right]=\left[\begin{array}{cc} 1 & 1\\ 1 & -1 \end{array}\right]\left[\begin{array}{c} x\left(t\right)\\ N\left(t\right) \end{array}\right], \end{array}$$

where *x*_*p*_*(t)*means*x(t)* add *N(t)* and *x*_*n*_*(t)*means*x(t)*subtract*N(t)*. Create many pairs (50 pairs in this study) of *x*_*p*_*(t)* and *x*_*n*_*(t)* by adding different white noise *N(t)*. Apply EMD to all *x*_*p*_*(t)* and *x*_*n*_*(t)* to extract the IMFs. Average all corresponding output IMFs to ensemble IMFs for reducing the influence of white noise.  Figure 2 shows the raw PPG signals and their related IMFs, for example (left column for a patient with lower severity of COPD; right column for a patient with higher severity of COPD). The IMF whose frequency approximates the original input signal will be determined as the main IMF (i.e., IMF3 in Figure 2).

The article "The Indices of Instantaneous Pulse Rate Variability Are Indicators for Daily Life Quality Assessment in Patients with COPD" was published in 2022. Journal: J Healthc Eng.

After finding out the main IMF, the normalized direct quadrature (NDQ) method is used for instantaneous frequency calculation [27]. Since main IMF is sinusoid, we can consider that main IMF is a cosine function *F(t)*. Therefore, the quadrature, sine function, can be calculated by

(6) $$\begin{array}{c} \text{sin}\emptyset \left(\text{t}\right)=\sqrt{1-{\text{F}}^{2}\left(\text{t}\right)}. \end{array}$$

Thus, the instantaneous phase can be obtained by arctan function:

(7) $$\begin{array}{c} \emptyset \left(\text{t}\right)=\text{arctan}\left(\frac{\text{sin}\emptyset \left(\text{t}\right)}{\text{F}\left(\text{t}\right)}\right). \end{array}$$

The instantaneous frequency *IF(t)* is obtained from the derivative of ∅*(t)*:

(8) $$\begin{array}{c} \text{IF}\left(\text{t}\right)=\emptyset^{\prime }\left(\text{t}\right). \end{array}$$

Finally, the instantaneous pulse rate *iPR(t)* is estimated by inversion of *IF(t)* in order to indicate the time series of heartbeat rhythm as RRi in HRV. Similar to the HRV power spectrum, the iPR(t) is transformed by fast Fourier transform (FFT) into frequency domain, and the power spectrum is calculated for further analysis.

(9) $$\begin{array}{c} {\text{S}}_{\text{xx}}\left(\text{f}\right)=\frac{{\text{FFT}}^{*}\left(\text{iPR}\left(\text{t}\right)\right){\times \text{FFT}}^{*}\left(\text{iPR}\left(\text{t}\right)\right)}{{\text{n}}^{2}}, \end{array}$$

where *S*_*xx*_*(f)* is the output power spectrum, ^*∗*^ denotes the complex conjugate, and *n* is the number of samples. The whole procedure of iPRV is shown in Figure 3.

### 2.5. Index Calculation

The standard bandwidth of low frequency (LF) band and high frequency (HF) band is 0.04 Hz to 0.15 Hz and 0.15 Hz to 0.4 Hz in HRV, respectively. In iPRV, the bandwidth of very high frequency (VHF) band is defined as 0.4 Hz to 0.9 Hz. Therefore, we can calculate the normalized LF (nLF), normalized HF (nHF), and normalized VHF (nVHF) as follows:

(10) $$\begin{array}{c} \text{nLF}=\frac{\text{LF}}{\text{TP}}*100\%, \end{array}$$

(11) $$\begin{array}{c} \text{nHF}=\frac{\text{HF}}{\text{TP}}*100\%, \end{array}$$

(12) $$\begin{array}{c} \text{nVHF}=\frac{\text{VHF}}{\text{TP}}*100\%, \end{array}$$

where TP is total power which can be calculated excluding VHF,

(13) $$\begin{array}{c} \text{TP}\left(\text{w}/\text{o VHF}\right)=\text{LF}+\text{HF}, \end{array}$$

or including VHF,

(14) $$\begin{array}{c} \text{TP}\left(\text{w}/\text{VHF}\right)=\text{LF}+\text{HF}+\text{VHF.} \end{array}$$

Therefore, two types of nLF and nHF exist. We use nLF^a^ and nHF^a^ to denote the normalized power calculated by TP(w/o VHF). nLF^b^, nHF^b^, and nVHF^b^ denote the normalized power calculated by TP(w/VHF). In addition, LF to HF ratio is calculated as

(15) $$\begin{array}{c} \text{LF}/\text{HF}=\frac{\text{LF}}{\text{HF}}*100\text{\%.} \end{array}$$

### 2.6. Statistical Analysis

Because of the small number of subjects and discrete grades of questionnaires, the nonparametric static method was performed in this study. Wilcoxon sign rank test was used for dependent variable distribution difference analysis. The results of Wilcoxon sign rank test were reported as mean ± standard deviation. The Spearman correlation coefficient was adopted to test the rank correlation between questionnaires and iPRV indices. Different from Pearson's correlation coefficient, which assesses the linear relationships, Spearman correlation measures the extent to which the trend between two variables is similar. It is not only suitable for comparing continuous variables, but also appropriate for assessing the relationship between discrete ordinal variables and continuous variables. The results of Spearman correlation coefficient were reported as r-values. The absolute r-values between 1 and 0.7, 0.7 and 0.4, 0.4 and 0.3, 0.3 and 0.2, and 0 and 0.2 indicate very strong, strong, moderate, weak, and no relationship, respectively. The *p*-value of Spearman correlation shows whether a significant correlation exists between two variables or not. All statistical analysis was conducted at a 95% level of significance and performed by using LabVIEW Probability and Statistics VI (v. 2018, National Instruments, Austin, USA).

The article "The Indices of Instantaneous Pulse Rate Variability Are Indicators for Daily Life Quality Assessment in Patients with COPD" was published in 2022. Journal: J Healthc Eng.

## 3. Results

The result of comparison between phase A and phase B indices is shown in Table 2. LF, HF, and VHF have significant difference between phase A and phase B (*p* < 0.05). The Spearman correlation coefficient result between questionnaires and iPRV indices is shown in Table 3. There was correlation of nLF^a^, nHF^a^, LF/HF, nLF^b^, and nHF^b^ with mMRC (*r* = 0.78, *r* = −0.78, *r* = 0.78, *r* = 0.62, and *r* = −0.61, respectively; *p* < 0.01 for nLF^a^, nHF^a^, and LF/HF; *p* < 0.05 for nLF^b^ and nHF^b^) in phase B. There was no correlation between iPRV indices and CAT in each phase.

The difference in mMRC between phase A and phase B had correlation with the difference in nLF^a^, nHF^a^, LF/HF, nLF^b^, and nHF^b^ (*r* = 0.60, −0.60, 0.63, 0.58, and −0.58, respectively; *p* < 0.05 for each). The change between phase A and phase B also had correlation between HF and VHF with CAT (*r* = −0.64 and *r* = −0.55, respectively; *p* < 0.05 for both).

In addition, the Spearman correlation coefficient was also performed between each subquestion of CAT and each iPRV index. The result is shown in Tables 4 and 5. For single phase, only LF in phase A had correlation with CAT7 (*r* = 0.58; *p* < 0.05). For the change between phase A and phase B, the correlation between the differences in each subquestion of CAT and the differences in iPRV indices is shown in Table 6, and Table 7 shows the difference score between phase B and phase A. CAT1 had correlation with HF and VHF (*r* = −0.61 and *r* = −0.54, respectively; *p* < 0.05 for both). CAT5 had correlation with LF (*r* = −0.53; *p* < 0.05). There was correlation of HF and VHF with CAT6 (*r* = −0.53 and *r* = −0.54, respectively; *p* < 0.05 for both). A correlation of HF and VHF with CAT7 was also found (*r* = −0.57 and *r* = −0.59, respectively; *p* < 0.05 for both). No correlation was found between iPRV indices and CAT2, CAT3, CAT4, and CAT8.

The article "The Indices of Instantaneous Pulse Rate Variability Are Indicators for Daily Life Quality Assessment in Patients with COPD" was published in 2022. Journal: J Healthc Eng.

## 4. Discussion

In this study, we aimed to compare the correlation between questionnaires and cardiovascular variability in COPD patients for finding how the cardiovascular activities affect the daily quality in patients with COPD.

### 4.1. iPRV Compared with mMRC and CAT

Four subjects' mMRC score did not change between the two phases; six subjects' mMRC score decreased in phase B, which means they feel better than before; four subjects' mMRC score increased in phase B, which means they breathe more hardly than before. For CAT score in phase B compared with phase A, twosubjects' scores did not change, ten subjects' scores decreased, and two subjects' scores increased, respectively (higher score in CAT means the condition is more serious.). Thirty subjects had the same trend of mMRC and CAT score in phase B compared with phase A (we assumed the score of mMRC and CAT increase or no change in phase B to be the same trend; the score of mMRC and CAT decrease or no change in phase B is also the same trend). Only one subject showed opposite trend (mMRC increase but CAT decrease in phase B). For the change in the iPRV indices, the index calculated with HF had significant correlation with these two questionnaires. The HF is modulated by vagus nerve and breathing [28]. This means that the scores of both questionnaires were possibly regulated by vagus nerve and breathing. However, only mMRC had significant correlation with the indices calculated with LF; only CAT had significant correlation with VHF. This can be interpreted as follows: the score of mMRC is more likely to be affected by the activity of SNS; the score of CAT is more likely to be affected by the peripheral regulation.

### 4.2. iPRV Result Compared with Subquestions of CAT

Each subquestion content of CAT is shown in Figure 4. For single phase, only CAT7 had significant correlation with LF in phase A. Most of subjects had higher score in CAT7 in phase A than that in phase B. This means that the worse quality of sleeping caused by pulmonary disease possibility has relation with SNS modulation. For the change in each subquestion of CAT between phase A and phase B, CAT1, CAT6, and CAT7 had significant correlation with HF and VHF, respectively. They are conditions for assessing breathing problems during daily life (CAT1: cough problem; CAT6: confidence to go outside despite having pulmonary disease; CAT7: sleeping quality). The peripheral response which is the possible meaning of change in VHF [24] and PNS may influence the scores of CAT1, CAT6, and CAT7. In addition, the change in CAT5 between phase A and phase B had significant correlation with LF. CAT5 assesses whether the quality of daily life at home is affected by lung problem or not. It may be influenced by the sympathetic nervous system. To sum up this paragraph, the problems of daily life caused by lung or breathing are more likely to be modulated by peripheral circulation and parasympathetic nervous system. Additionally, the quality of activity of patients at home is more likely to be affected by sympathetic nervous system. Trying to adjust the activity of ANS and peripheral circulation may make patients with COPD feel better in their daily life.

The article "The Indices of Instantaneous Pulse Rate Variability Are Indicators for Daily Life Quality Assessment in Patients with COPD" was published in 2022. Journal: J Healthc Eng.

A previous study showed that functional capacity was negatively associated with PNS in COPD exacerbation [18]. Though the subjects of this study were not assessed as to whether they are in COPD exacerbation or not and even most of subjects in phase B had lower scores in mMRC and CAT, which means their condition of COPD is better than before, we still found that the breathing problem, which may be caused by functional capacity, in daily life of patients with COPD had relation with the modulation of PNS.

### 4.3. Related Work Comparison

Camillo et al. compared the relation between HRV indices and different disease characteristics [17]. They measured 3 questionnaires (MRC, Saint George Respiratory Questionnaire (SGRQ) which evaluates the health-related quality of life, and London Chest Activity of Daily Living (LCADL) scale which assesses the activities limit in daily life), muscle function, and physical activity in daily life using SenseWear. They found that the time domain index standard deviation of the N-N intervals (SDNN) had higher significant correlation with LCADL and physical activity in daily life, especially total daily energy expenditure. LF/HF also had significant correlation with total daily energy expenditure in their findings. Additionally, LF/HF had higher significant correlation with the muscle function (quadriceps force, biceps force, and maximal expiratory pressures (MEP)) in their research. However, LF/HF had higher significant correlation with mMRC in our study, which was not found in the previous study. One possible explanation is that we measured the mMRC instead of MRC. In addition, the patients in our study had lower score of mMRC. This means that LF/HF would influence the patients' breathing during exercise in lighter condition of COPD. Moreover, the previous study showed that LF/HF had relation with MEP which possibly affects the score of mMRC. Some studies also showed reduced balance and coordination in patients with COPD compared to healthy people [29]. This may have relationship with MEP and ANS activities. However, it still needs more research to be validated.

The article "The Indices of Instantaneous Pulse Rate Variability Are Indicators for Daily Life Quality Assessment in Patients with COPD" was published in 2022. Journal: J Healthc Eng.

## 5. Limitations

This study had some limitations. Some spirometry results were missing in phase B. Therefore, we cannot compare the lung function change with the questionnaires and iPRV indices. Only VC and V_t_ measured during the first minute of experiment can be indicated. However, no significant correlation between these two indices and iPRV indices or questionnaires was found. The duration of signal used for analysis is short. Though some research showed that iPRV has the potential to be a short term evaluation by using instantaneous frequency technique [30], it still needs to be examined in the patients with COPD. For further research, a larger number of subjects are necessary to confirm the reliability of iPRV analysis. In addition, to compare the different breathing maneuver and analysis, the cardiovascular variability can be helpful information for pulmonary rehabilitation.

## 6. Conclusion

In conclusion, this study showed the change in iPRV indices while the condition of COPD was improvement (score of mMRC or CAT decrease) or exacerbation (score of mMRC or CAT increase). LF/HF was related to the change of mMRC, which assesses the breathing ability when exercising. HF and the novel index, VHF calculated by iPRV, were related to the change of CAT, which assess the quality of daily life of patients with COPD. According to the ANS activity and peripheral response, the result showed that the interaction between cardiovascular activity and respiratory mechanism affects daily life quality in patients with COPD. Increase in LF or decrease in HF and VHF would lead to poorer quality of daily life in patients with COPD. For quality of daily life improvement, the ANS regulation and peripheral response in patients with COPD should be taken care of in rehabilitation or therapy program. The PPG is an easy to use instrument in daily life. Most of smart phones/watches can detect PPG waveform. The iPRV indicators are useful for daily healthcare of patients with COPD. The further research is to examine which breathing type can regulate the ANS and peripheral response to suitable status to make patients with COPD have better quality of daily life.

## Figures and Tables

**Figure 1:** The demonstration of RRi (left top), HRV spectrum (right top), iPR series (left bottom), and iPRV spectrum (right bottom).

**Figure 2:** The raw PPG and IMFs compared between patients with different severities of COPD. Score of mMRC = 1 and CAT = 2 (left column); score of mMRC = 4 and CAT = 34 (right column).

**Figure 3:** The demonstration of iPRV procedure.

The article "The Indices of Instantaneous Pulse Rate Variability Are Indicators for Daily Life Quality Assessment in Patients with COPD" was published in 2022. Journal: J Healthc Eng.

**Figure 4:** The CAT questionnaire. Source: Jones et al. [3].

**Table 1:** Basic information of subjects.

Variables	COPD (*n* = 14)	
	Phase A	Phase B
Age (years)	75 ± 9.5	75 ± 9.5
Males, *n* (%)	12 (86)	12 (86)
Height (cm)	161.00 ± 7.98	160.46 ± 7.60
Weight (kg)	62.8 ± 14.17	62.4 ± 14.98
BMI	24.21 ± 4.85	24.09 ± 4.97
Body fat (%)	24.71 ± 6.18	24.89 ± 6.29
mMRC	1.86 ± 0.83	1.5 ± 0.82
CAT	13.50 ± 5.22	10.36 ± 6.80
BR (breaths/min)	19.01 ± 5.70	19.24 ± 4.82
PR (beats/min)	86.50 ± 15.74	82.45 ± 17.31
V_T_ (L)	0.68 ± 0.36	0.66 ± 0.67
VC (L)	2.16 ± 0.84	2.02 ± 0.36

BMI: body mass index; BR: breathing rate; PR: pulse rate; VT: tidal volume; VC: vital capacity.

**Table 2:** iPRV values in two phase.

Phase	LF	HF	VHF	nLF^a^	nHF^a^	LF/HF	nLF^b^	nHFb	nVHF^b^
A	0.37 ± 1.09	0.67 ± 2.00	1.98 ± 6.57	37.30 ± 18.7	62.70 ± 18.70	82.42 ± 89.20	16.33 ± 13.90	23.63 ± 8.77	60.05 ± 15.31

B	1.54 ± 2.63^*∗*^	3.13 ± 7.20^*∗*^	4.77 ± 9.36^*∗*^	35.03 ± 16.84	64.97 ± 16.84	65.37 ± 48.17	15.79 ± 8.27	29.61 ± 14.08	54.59 ± 15.16

^*∗*^ *p* value< 0.05 compared with phase A by Wilcoxon sign rank test.

**Table 3:** Correlation between iPRV indices and questionnaires.

Variables	LF	HF	VHF	nLF^a^	nHF^a^	LF/HF	nLF^b^	nHFb	nVHF^b^
*Phase A*									
mMRC	0.09	−0.02	−0.07	0.32	−0.32	0.32	0.31	−0.18	−0.08
CAT	0.47	0.31	0.20	0.11	−0.11	0.11	0.12	0.06	−0.26

*Phase B*									
mMRC	0.15	0.09	0.07	0.78^*∗∗*^	−0.78^*∗∗*^	0.78^*∗∗*^	0.62^*∗*^	−0.61^*∗*^	0.19
CAT	−0.13	−0.18	−0.20	0.28	−0.28	0.28	0.17	−0.21	0.02

*B-A*									
mMRC	0.03	−0.22	−0.1^*∗*^	0.60^*∗*^	−0.60^*∗*^	0.63^*∗*^	0.58^*∗*^	−0.58^*∗*^	0.18
CAT	−0.3	−0.64^*∗*^	−0.55^*∗*^	0.39	−0.39	0.50	0.39	−0.53	0.19

^*∗*^ *p*-value< 0.05. ^*∗∗*^*p*-value<0.01. B-A difference score of mMRC was −0.36 ± 1.34 and CAT was −3.14 ± 6.54.

**Table 4:** Correlation between iPRV indices and each subquestion of CAT in phase A.

Variables	LF	HF	VHF	nLF^a^	nHF^a^	LF/HF	nLF^b^	nHFb	nVHF^b^
CAT1	0.41	0.37	0.23	0.01	−0.01	0.01	0.26	0.21	−0.38
CAT2	0.33	0.17	0.09	0.08	−0.08	0.08	0.11	−0.08	−0.20
CAT3	0.24	0.26	0.22	−0.06	0.06	−0.06	0.12	0.49	−0.33
CAT4	−0.12	−0.21	−0.28	0.22	−0.22	0.22	0.15	−0.36	0.11
CAT5	0.03	0.12	0.08	0.02	−0.02	0.02	0.04	0.01	0.04
CAT6	−0.18	−0.46	−0.41	0.32	−0.32	0.32	0.02	−0.38	0.02
CAT7	0.58^*∗*^	0.49	0.40	0.00	0.00	0.00	0.07	0.05	−0.21
CAT8	0.34	0.36	0.39	−0.17	0.17	−0.17	−0.13	0.31	−0.09

^*∗*^ *p*-value< 0.05.

**Table 5:** Correlation between iPRV indices and each subquestion of CAT in phase B.

Variables	LF	HF	VHF	nLF^a^	nHF^a^	LF/HF	nLF^b^	nHFb	nVHF^b^
CAT1	−0.03	−0.06	−0.04	0.28	−0.28	0.28	0.24	−0.31	−0.01
CAT2	−0.03	−0.03	−0.04	0.16	−0.16	0.16	0.01	−0.27	0.13
CAT3	0.12	0.06	0.09	0.05	−0.05	0.05	0.14	−0.28	−0.11
CAT4	0.06	0.08	0.01	−0.01	0.01	−0.01	−0.11	0.30	−0.07
CAT5	−0.04	−0.04	0.00	0.20	−0.20	0.20	−0.04	−0.20	0.35
CAT6	−0.25	−0.35	−0.30	0.37	−0.37	0.37	0.36	−0.31	0.04
CAT7	−0.33	−0.41	−0.45	0.30	−0.30	0.30	0.30	−0.13	−0.08
CAT8	−0.29	−0.37	−0.41	0.32	−0.32	0.32	0.23	−0.15	−0.05

^*∗*^ *p*-value< 0.05.

The article "The Indices of Instantaneous Pulse Rate Variability Are Indicators for Daily Life Quality Assessment in Patients with COPD" was published in 2022. Journal: J Healthc Eng.

**Table 6:** Correlation between iPRV indices and each subquestion of CAT in phase B–phase A.

Variables	LF	HF	VHF	nLF^a^	nHF^a^	LF/HF	nLF^b^	nHFb	nVHF^b^
CAT1	−0.50	−0.61^*∗*^	−0.54^*∗*^	0.05	−0.05	0.10	0.14	−0.25	0.12
CAT2	−0.12	−0.39	−0.28	0.16	−0.16	0.24	0.12	−0.42	0.28
CAT3	0.09	0.02	0.03	0.15	−0.15	0.18	0.04	−0.27	0.17
CAT4	−0.07	−0.16	−0.10	0.07	−0.07	0.12	0.12	−0.15	0.25
CAT5	−0.53^*∗*^	−0.29	−0.29	−0.07	0.07	−0.11	−0.11	−0.25	0.37
CAT6	−0.32	−0.53^*∗*^	−0.54^*∗*^	0.42	−0.42	0.52	0.24	−0.43	0.13
CAT7	−0.35	−0.57^*∗*^	−0.59^*∗*^	0.27	−0.27	0.32	0.33	−0.18	−0.23
CAT8	0.12	−0.11	−0.05	0.09	−0.09	0.14	0.13	−0.23	0.03

^*∗*^ *p*-value< 0.05.

**Table 7:** Score difference between phase B and phase A.

Variables	B-A difference
CAT1	−0.71 ± 1.94
CAT2	−0.07 ± 1.54
CAT3	0.14 ± 1.56
CAT4	−1.07 ± 1.98
CAT5	0.07 ± 0.47
CAT6	−0.71 ± 1.54
CAT7	−0.36 ± 2.24
CAT8	−0.43 ± 1.02

## Data Availability

The PPG data used to support the findings of this study are available from the corresponding author upon request. However, for protecting the rights and privacy of each subject, all who want to access our data should provide the IRB approval.
